# An Artificial Neural Network Based Analysis of Factors Controlling Particle Size in a Virgin Coconut Oil-Based Nanoemulsion System Containing Copper Peptide

**DOI:** 10.1371/journal.pone.0157737

**Published:** 2016-07-06

**Authors:** Shazwani Samson, Mahiran Basri, Hamid Reza Fard Masoumi, Emilia Abdul Malek, Roghayeh Abedi Karjiban

**Affiliations:** Department of Chemistry, Faculty of Science, Universiti Putra Malaysia, UPM Serdang, Selangor, Malaysia; VIT University, INDIA

## Abstract

A predictive model of a virgin coconut oil (VCO) nanoemulsion system for the topical delivery of copper peptide (an anti-aging compound) was developed using an artificial neural network (ANN) to investigate the factors that influence particle size. Four independent variables including the amount of VCO, Tween 80: Pluronic F68 (T80:PF68), xanthan gum and water were the inputs whereas particle size was taken as the response for the trained network. Genetic algorithms (GA) were used to model the data which were divided into training sets, testing sets and validation sets. The model obtained indicated the high quality performance of the neural network and its capability to identify the critical composition factors for the VCO nanoemulsion. The main factor controlling the particle size was found out to be xanthan gum (28.56%) followed by T80:PF68 (26.9%), VCO (22.8%) and water (21.74%). The formulation containing copper peptide was then successfully prepared using optimum conditions and particle sizes of 120.7 nm were obtained. The final formulation exhibited a zeta potential lower than -25 mV and showed good physical stability towards centrifugation test, freeze-thaw cycle test and storage at temperature 25°C and 45°C.

## 1. Introduction

Aging is a process defined as a progressive deterioration of the physiological functions of skin [1]. This process occurs in all living tissues especially skin and this causes wrinkles, sagging, pigmented spots and dryness. Two types of aging; intrinsic (genetic factors) and extrinsic (environmental factors) occur due to passage of time [2] and exposure to ultraviolet radiation, respectively. The first type causes irreversible degeneration of skin tissue, loss of skin thickness and elastic tissue and reduction in the number of dermal fibroblasts, whereas the latter leads to the formation of coarse and rough skin with deep lines, wrinkles and hyperpigmentation in the skin. In order to reduce the skin problems caused by aging, compounds having specific properties such as antioxidant or rejuvenating abilities could be used.

Antioxidants are believed to play a role in preventing cells from oxidative stress caused by the overproduction and accumulation of reactive oxygen species (ROS) [3]. These compounds neutralize free radicals by pairing with oxygen in the destabilization process [4]. On the other hand, cosmeceutical peptides are important in many natural processes involving skin care. The peptide chain is capable of regulating the production of extracellular matrix components such as fibroblast cells [5]. One of the more well-known cosmeceutical peptides is the copper peptide (copper complex of human tripeptide, glycyl-l-histidyl-l-lysine-Cu) which possesses not only anti-aging and reparative properties but also can function as an antioxidant [6,7]. It works by scavenging toxic free radicals and thereby reduces oxidative damage, modulates copper level in skin cells and facilitates cellular interaction with the extracellular matrix giving it the ability to exhibit excellent reparative, protective and rejuvenating properties on skin [6].

The amount of peptides [8] that can be delivered into the skin through oral supplementation is limited due to the physiological processes related to active absorption, stability and solubility. Therefore, topical application has the added advantage of targeting the antioxidants and peptides to the specific area of skin which requires protection. Nanoemulsions have been used to enhance the penetration and permeability of active ingredients through the *stratum corneum* [9] due to the small size of the particles in the nanoemulsion (20–200 nm). Nanoemulsions have also become attractive for applications in both pharmaceutical and cosmetic industries due to their high kinetic stability [10, 11], non-toxic and non-irritant properties and also their suitability for efficient delivery of active compounds through the skin [11]. For topical use, the small size of droplets in nanoemulsions allows them to be deposited uniformly on the skin thus enhancing their penetration [12].

Virgin coconut oil that was used in this study is oil obtained from the fresh and mature kernel of coconuts without undergoing any chemical refining. It is a saturated fat consisting mainly of medium chain fatty acids with several functions including medical, pharmaceutical, and cosmetic and in dietary oils [13]. In terms of cosmetic usage, virgin coconut oil has been reported to have skin moisturizing properties and was found to be useful for skin applications [14]. The medium chain triglyceride and the monoglyceride content of the oil contribute to its antibacterial properties [15]. The oil also demonstrated excellent antioxidant activity due to its phenolic content [16].

In order to prepare a suitable nanoemulsion for the topical delivery of copper peptide, optimization of the composition needs to be carried out first. The optimization of the mixture composition to obtain a product with the required characteristics is one of the common issues in the pre-formulation of cosmetic products. There are several statistical techniques used for the optimization of mixture compositions and processing parameters to obtain desirable properties including the response surface methodology [17–20], Box Behnken, D-optimal mixture design [21–23] and artificial neural network (ANN) [24–30]. In this study, ANN was utilized to optimize the composition of the VCO nanoemulsion by considering particle size as the response parameter. ANN is able to correlate the complex relationship between system parameters without fully understanding the system’s mechanism and has been applied in the modeling of various complex system parameters [31]. To the best of our knowledge, there are no reported studies on the optimization of VCO based nanoemulsions using ANN and only a few reports are available on the optimization of cosmetic products using this type of mathematical tool.

Hence, in this work, we report the use of ANN to model the relationship between nanoemulsion composition (oil, emulsifier, xanthan gum and water) and particle size and the successful formulation of a VCO nanoemulsion containing an active (copper peptide) using the optimum conditions as predicted by the model.

## 2. Materials and Methods

### 2.1. Materials

Copper peptide was obtained from GL Biochem Ltd Shanghai, China. Virgin coconut oil, xanthan gum, Tween 80 (Polyoxyethylenesorbitan monostearate) and Pluronic F68 (PF68) were purchased from Sigma-Aldrich, St Louis, USA. Phenonip was procured from Bramble Berry Bellingham, USA. Water was deionized using a Milli-Q filtration system.

### 2.2. Formation of VCO based nanoemulsion

The preparation of oil phase was carried out by mixing T80:PF68 (40:1) and VCO while for the aqueous phase, xanthan gum was added into deionized water. The oil and aqueous phase were initially heated separately until all the ingredients dissolved. Using a homogenizer, the aqueous phase was added drop wise into the oil phase until complete. The final mixture was homogenized for 3 hours using an overhead stirrer. The emulsion obtained was further subjected to a high shear homogenizer for 10 minutes at 15000 rpm. Phenonip (0.7% w/w) was added as an anti-microbial agent.

### 2.3. Preliminary study on the different process parameters

This experiment was carried out following the method described in Section 2.2. The amount of mixed surfactant, VCO and xanthan gum used were 15%, 10%, and 0.5% w/w respectively. The final mixture was homogenized for 3 hours using an overhead stirrer. The emulsion obtained was further subjected to a high shear homogenizer at different shear time (5, 10, 15, 20 min) at 10000 rpm and different shear speed (5000, 10000, 15000 rpm) at 10 min mixing time. Phenonip (0.7% w/w) was added as an anti-microbial agent.

### 2.4. Formation of VCO based nanoemulsion containing copper peptide

The nanoemulsion was prepared following the method described in Section 2.2. After the addition of active matter (copper peptide 0.003% w/w) into the pre-mixed emulsion, the final mixture was homogenized for 3 hours using an overhead stirrer. The emulsion obtained was further subjected to a high shear homogenizer for 10 minutes at 15000 rpm. Phenonip (0.7% w/w) was added as an anti-microbial agent.

### 2.5. Particle size measurements

Particle size was determined by a dynamic light scattering technique, scattered at an angle of 173° at 25°C. The measurements were carried out using a Zetasizer (Nano ZS, Malvern Instrument Ltd., UK). Intensity distribution was used for the measurement of mean average (z-average) droplet size. The samples were diluted with deionized water in order to avoid multiple scattering effects. Measurements were taken three times.

### 2.6. Artificial neural network (ANN) software tool and data sets

The modeling and optimization of the VCO nanoemulsion were performed using the NeuralPower software version 2.5. This software operates *via* a graphical user interface (GUI) which helps the user to load the training and testing sets, design the network architecture, select the training algorithm and generate the individual models for each output variable, all in one single operation [24]. In order to design the experiments, the level of effective input variables were considered which included VCO (10–20%, w/w), T80:PF68 (10–15%, w/w), xanthan gum (0.5–1.0%, w/w) and water (64.008–79.291%, w/w) while particle size was taken as the response. Table 1 depicts the experimental data with actual and predicted values of particle size used for ANN design. A total of 26 experiment points were randomly divided into 3 data sets; training set (16 points), testing set (6 points) and validation set (4 points). Training data was used to train neural network weights while testing data was to confirm the robustness of the network parameters besides avoiding the over fitting by controlling errors [32]. The validation set was used to check the adequacy of the final model obtained using the software

**Table 1:** The experimental design consists of training, testing and validation data sets; each row indicates an experiment while the columns present the composition of the VCO nanoemulsions.

Run No.	VCO	T80:PF68	Xanthan Gum	Water	Actual Particle size (nm)	Predicted Particle size (nm)
**Training set**						
1	10.003	10.000	0.706	79.291	138.95	142.62
2	10.089	15.000	0.503	74.408	137.25	123.79
3	20.000	10.435	0.610	68.954	617.50	622.63
4	20.000	10.435	0.610	68.954	628.73	622.63
5	15.168	13.202	0.757	70.873	161.23	171.65
6	19.902	10.729	1.000	68.369	427.22	430.09
7	17.696	14.064	0.500	67.740	167.40	160.14
8	19.994	15.000	0.998	64.008	299.57	296.63
9	10.089	15.000	0.503	74.408	126.60	123.79
10	17.743	10.121	0.977	71.160	453.52	450.43
11	12.822	10.000	0.502	76.676	148.00	149.37
12	13.156	12.532	0.500	73.812	135.40	132.64
13	19.994	15.000	0.998	64.008	295.23	296.63
14	12.773	14.996	1.000	71.231	136.00	132.03
15	10.003	10.000	0.706	79.291	145.27	142.62
16	20.000	14.994	0.502	64.505	139.37	145.07
**Testing set**						
1	13.500	12.532	0.706	72.762	155.32	155.22
2	14.000	14.500	0.570	70.430	130.68	131.78
3	14.500	14.500	0.570	69.930	134.87	134.20
4	15.500	14.500	0.570	68.930	140.65	140.47
5	11.000	12.532	0.706	75.762	139.90	139.73
6	10.000	15.000	0.500	74.500	122.90	123.50
**Validation set**						
1	11.000	12.532	0.706	75.262	140.50	136.90
2	10.000	15.000	0.5	74.500	124.60	122.30
3	10.000	15.000	0.5	74.500	121.70	122.30

### 2.7. ANN architecture

ANN is an information-processing paradigm which is based on biological nervous systems such as the human brain [33]. It is a computing system made up of units which are a highly interconnected set of simple information processing elements similar to neurons. These neurons gather inputs from single and multiple sources and provide output in accordance with a predetermined non-linear function [30]. Artificial neural network is a useful tool for the optimization of nanoemulsions as the preparation of nanoemulsions depends on the combination of several parameters affecting the properties, especially those that involve complex and highly nonlinear relationships [28]. In this work, the ANN model used for the problem-fitting purpose was a multilayer feed-forward neural network containing three layers. The architecture of ANN consists of an input layer, a hidden layer and an output layer. The artificial neurons or nodes are the basic processing elements of neural networks. These neurons are connected to each other to transmit signals from the input layer passing through the hidden layer to the output layer [27]. In order to select the optimum number of neurons in the hidden layer, a trial and error approach was utilized. This was done by starting from a minimum number of neurons and then was gradually increased depending on the nature of the problem. It is very important to determine the number of neurons in the hidden layer as it will affect the performance of the network [34]. Each neuron in the hidden or output layer, acting as a summing junction, combines and modifies the inputs from the previous layer [35–36, 24]. This is done using the following equation:

$$y_{i}=\sum_{j=1}^{i}x_{i}w_{ij}+b_{j}$$ (1)

where *y*_*i*_ is the net input to node *j* in the hidden or output layer, *x*_*i*_ as the inputs to node *j* while *w*_*ij*_ are the weights which represents the strength of connection between *ith* node and *jth* node, *i* is the number of nodes and *b*_*j*_ is the bias related to node *j*. Each neuron consists of a transfer function which is responsible for the transformation of an input into an output [24]. There are several types of transfer functions used in literature such as the Tanh transfer function [28,33] and sigmoid transfer function [24,34]. In this work, the sigmoidal transfer function was used for both hidden and output layers. The sigmoid (logistic) function (Eq 2) was applied on the weighted summed of neuron’s input in the hidden layer before transferring to output layer.

$$\text{f}\left(\text{x}\right)=\frac{1}{1+\text{ exp}\left(-\text{x}\right)}$$ (2)

where, *f(x)* is the activation function.

Several types of learning algorithms were used in this work since it is difficult to determine which learning algorithm will be more efficient for a given problem [24]. These include incremental backpropagation (IBP), batch backpropagation (BBP), quick propagation (QP), genetic algorithm (GA) and Levenberg-Marquardt backpropagation (LM).

### 2.8. Evaluation of model predictability

The mean squared error (MSE) or root mean squared error (RMSE) as in Eq 3 was used in this study to perform a supervised training. This measurement was performed in order to evaluate the ANN output error between the actual and predicted outputs.

$$RMSE={\left(\frac{1}{n}\;\sum_{i=1}^{n}{\left(y_{i}-y_{di}\right)}^{2}\right)}^{1/2}$$ (3)

where *n*, *y*_*i*_ and *y*_*di*_ are the number of points, predicted values and actual values respectively. The learning process, in which the aim was to find the weights for minimizing RMSE, was carried out with an algorithm until the minimum RMSE (topology) was obtained. The topology was repeated several times to prevent random correlation caused by the random initialization of weights. The obtained topology with the lowest RMSE was selected and compared with other nodes’ topologies. Finally, the topologies of different algorithms were compared and the optimum model was selected based on maximum R^2^ (Eq 4), minimum RMSE and AAD (Eq 5).

$$R^{2}=1-\frac{\sum_{i=1}^{n}{\left(y_{i}-\;y_{di}\right)}^{2}}{\sum_{i=1}^{n}{\left(y_{di}-\;y_{m}\right)}^{2}}$$ (4)

$$AAD=\frac{1}{n}\;\sum_{i=1}^{n}\frac{\left|y_{i}-\;y_{di}\right|}{y_{di}}$$ (5)

where the number of points are represented by *n*,and *y*_*i*_ and *y*_*di*_ are predicted and actual values respectively and *y*_*m*_ is the average of the actual values.

### 2.9. Zeta potential analysis

Zeta potential analysis was carried out using a Zetasizer (Nano ZS, Malvern Instrument Ltd., UK) at room temperature. Samples were diluted with deionized water prior to measurement. The calculation of zeta potential was done based on the measurement of the electrophoretic mobility of dispersed particles in a charged field.

### 2.10. Stability study

This test was carried out to predict the long term physical stability of the nanoemulsions. For storage stability, VCO nanoemulsions were kept at two storage temperatures (25°C and 45°C). The physical appearances of the formulations (no sedimentation, creaming, coalescence and phase separation) were observed within 3 months. Samples were also subjected to centrifugal force at 4500 rpm for 15 min. The freeze-thaw cycle test was conducted by alternately keeping the formulations at 4°C and 25°C for 24 h for 6 days. Observation of phase changes was recorded for each day.

## 3. Results and Discussion

### 3.1. Preliminary study

The preliminary study on the different process parameters was carried out to find out the optimum shear time and shear speed that could produce nanoemulsion with minimum particle size. The effect of shear time on particle size is as depicted in Table 2. The homogenization time indicates the time spend by the emulsion in the homogenizer during the mixing process for the oil and aqueous phases. The results obtained showed that higher particle size was produced at low level of homogenization speed (5 min) due to the insufficient residence time of the surfactant molecules to allow their adsorption onto the entire droplet surface available during the homogenization process. Smaller particle size was observed at shear time of 10 min and became nearly constant at time greater than 10 min. On the other hand, increased in homogenization speed gave lower particle size (Table 3). The mixing force involved in the breakup of larger droplets into smaller one was the mechanical impact against the wall influenced by the high fluid acceleration as well as the shear stress in the gap between the rotor and the stator caused by rapid rotation of the stator. At lower shear speed, the mixing energy was insufficient giving larger particle size.

**Table 2:** Particle size (nm) of nanoemulsion at different shear time (min).

Shear time (min)	Particle size (nm)
5	131.07 ± 2.57
10	125.50 ± 1.05
15	125.80 ± 0.99
20	125.53 ± 1.05

**Table 3:** Particle size (nm) of nanoemulsion at different shear speed (rpm).

Shear speed (rpm)	Particle size (nm)
**5000**	138.90 ± 0.70
**10000**	125.50 ± 1.05
**15000**	114.13 ± 0.58

### 3.2. The topologies of the algorithm

Optimization of ANN topology is the main step in the development of an ANN model. In this work, the examined neural network included four nodes in the input layer (VCO, T80:PF68, xanthan gum and water) and one node in the output layer (particle size, nm). The number of nodes in the hidden layer was determined by performing a series of topologies with varied node numbers from 1 to 15 for each algorithm involved. Model learning for testing data set was carried out to find the minimum value of RMSE which acts as the error function. The learning process was repeated 10 times for each node to prevent random correlation caused by random initialization of the weight [32]. This step was performed similarly for QP, IBP, BBP, GA, and LM algorithms to determine the optimum topology for each algorithm. The node with minimum value of RMSE was selected and plotted against the nodes of the algorithms’ hidden layer as shown in Fig 1.

**Fig 1:** The selected RMSE vs. node number of the VCO nanoemulsions network’s hidden layer for IBP, BBP, QP, GA and LM. The lowest RMSE belongs to node number 5 (IBP), 5 (BBP), 8 (QP), 11 (GA), and 7 (LM).

One node with the lowest RMSE among 15 topologies from each algorithm involved was selected as the best topology and compared. The selected topologies were 4-5-1 for both IBP and BBP, 4-8-1 for QP, 4-11-1 for GA and 4-7-1 for LM. As can be seen from Fig 2, the lowest RMSE amongst other topologies was shown by GA-4-11-1. However, further comparison between the performance data of the topologies was carried out to select the best model for the ANN.

**Fig 2:** Scatter plot of predicted particle size (nm) values *versus* actual conversion (%) values by using five algorithms for the testing data set.

### 3.3. Model Selection

The values of RMSE, R^2^ and AAD were evaluated for the topologies IBP-4-5-1, BBP-4-5-1, QP-4-8-1, GA-4-11-1 and LM-4-7-1. A graph of predicted versus actual values of particle size was plotted for both testing set and training set data to determine the R^2^ value. Fig 2 showed that the highest R^2^ for the testing data set (0.9973) was presented by topology GA-4-11-1 with R^2^ value for training data set (Fig 3) equal to 0.9989. The AAD of the testing and training data sets for the topologies are tabulated in Table 4. From this table, the lowest AAD was also shown by topology GA-4-11-1. Therefore, GA-4-11-1 was selected as the final optimum model for the optimization of VCO nanoemulsions since it showed minimum RMSE and AAD as well as maximum R^2^ when compared to other topologies. Fig 4 shows the final model (network GA-4-11-1) which consists of input, hidden and output layers.

**Fig 3:** Scatter plot of predicted particle size (nm) values *versus* actual particle size (nm) values by using five algorithms for the training data set.

**Fig 4:** Schematic representation of a multilayer perception feedforward network of ANN based on GA consisting of four inputs, one hidden layer with 11 nodes and one output.

**Table 4:** The performance data of the optimized topologies, IBP-4-5-1, BBP-4-5-1, QP-4-8-1, GA-4-11-1, and LM-4-17-1 of the VCO nanoemulsions.

Learning algorithm	Architecture	Training data			Testing data			Validation data		
		RMSE	R^2^	AAD	RMSE	R^2^	AAD	RMSE	R^2^	AAD
**LM**	4-7-1	3.0532	0.9997	0.9873	5.5678	0.9830	3.3252	7.1774	0.9795	4.8400
**IBP**	4-5-1	3.8222	0.9995	1.7084	4.1293	0.8940	2.7950	5.8020	0.9795	4.3586
**BBP**	4-5-1	5.2896	0.999	2.4601	3.7333	0.9158	2.2599	5.4893	0.9795	3.6836
**QP**	4-8-1	7.2797	0.9982	3.2924	1.9688	0.9632	1.2992	1.9221	0.9795	1.1897
**GA**	4-11-1	5.7036	0.9989	2.6172	0.5902	0.9973	0.3568	2.4907	0.9795	1.6337

### 3.4. Model validation

Validation of the selected model was performed to check the adequacy of the final model. The coefficient of determination, R^2^ between the observed and predicted particle size for 4 individual sets of the validation data was quite high with a value of 0.9795 (graph not shown), showing that the model obtained was quite significant.

### 3.5. Importance of the effective variables

Fig 5 depicts the importance in percentage of input variables on the particle size of VCO nanoemulsions. All selected variables were strongly influential on the particle size which indicated that any of the variables in this study could not be neglected for the composition analysis. As demonstrated in Fig 5, the most important factor was the xanthan gum content (28.56%). This was followed by T80:PF68 (26.9%), VCO (22.8%) and water (21.74%).

**Fig 5:** The relative importance of of input variables VCO, T80:PF68, xanthan gum, and water in the VCO nanoemulsion.

### 3.6. Optimum VCO nanoemulsions

A desirable formulation attained by preparing the VCO nanoemulsions with specific conditions is referred to as the optimum formulation. The optimized formulation labeled as Opt-VCO in this work has the composition of VCO, T80:PF68, xanthan gum and water at 10% w/w, 15% w/w, 0.867% w/w and 74.133% w/w, respectively as tabulated in Table 5. The predicted particle size for the optimum formulation was 124.16 nm. There was no significant difference between the actual and predicted values of particle size for the optimum formulation with an RSE value of 1.18%.

**Table 5:** The predicted and actual response values for the optimized formulation.

(VCO) %	(T80:PF68) %	(Xanthan Gum) %	(Water) %	Actual Particle Size (nm)	Predicted Particle Size (nm)	RSE %
10	15	0.867	74.133	122.70	124.16	1.18

### 3.7. Formulation of VCO nanoemulsions containing copper peptide

For the preparation of VCO nanoemulsions containing the active, copper peptide was incorporated into the Opt-VCO formulation. Table 6 shows the particle size of the VCO nanoemulsion containing 0.003% (w/w) copper peptide (VCOCP). There was no significant difference observed between the particle size of the optimum formulation and formulation containing the active where the difference was around 2.00 nm. The resulting VCOCP which has small particle size could hence be used as cosmeceutical for anti-aging purpose since the nano-sized emulsion can enhance the delivery or penetration of copper peptide through the skin.

**Table 6:** Response value for Opt-VCO and VCOCP.

Response	Opt-VCO	VCOCP
Particle size (nm)	122.70	120.70

### 3.8. Zeta potential of the final formulations

Measurement of zeta potential is important to predict the long term stability of formulations as well as to understand the state of the surface of the nanoparticles [37]. This parameter is not only responsible for the stability of colloidal dispersions but it provides an indication of the degree of repulsion between particles with identical charge in the dispersion [38]. Nanoemulsions with a high degree of stability are characterized as having zeta potential values higher than +25 mV or lower than -25 mV. Table 7 shows the zeta potential values of Opt-VCO and VCOCP. A low zeta potential (less than -25mV) is indicative of a good stability for all formulations.

**Table 7:** Zeta potential (mV) of the optimum VCO nanoemulsion and VCO nanoemulsion containing active compound.

Nanoemulsion systems	Zeta potential (mV)
**Opt-VCO**	-32.63 ± 1.27
**VCOCP**	-32.70 ± 2.16

### 3.9. Stability study

This test was carried out to predict the stability of cosmetic products when exposed to different situations that may occur under market conditions [38]. Therefore, Opt-VCO and VCOCP were subjected to various extreme storage conditions to evaluate the ability of samples to withstand the conditions over a period of time. Under centrifugation, the rate of creaming or sedimentation (phase separation) can be accelerated. Centrifugation test is used to predict the shelf life under normal storage conditions by observing the creaming or coalescence of the dispersed phase [39]. Table 8 shows that both the formulations exhibited no phase separation after centrifugation at 4500 rpm for 15 min. This was a positive indication of the stability of the formulations, if phase separation occurs; all the physical and chemical properties of the formulations will be affected.

**Table 8:** Centrifugation test.

Nanoemulsion systems	Observation
**Opt-VCO**	Stable
**VCOCP**	Stable

For the freeze-thaw cycling test; Opt-VCO and VCOCP were found to be stable (homogenous) after 6 days as depicted in Table 9. When the samples freeze, the oil droplets can be segregated from the emulsion by the crystallized ice particles and this leads to the disruption of the lipid film surrounding the droplets. These droplets can be melted and coalesced between approaching droplets when subjected to thaw leading to phase separation. All the formulations were observed to be in one phase even when temperatures were drastically changed. The stability of the formulations was probably due to the incorporation of xanthan gum. Xanthan gum is expected to be able to reduce both the re-association of oil droplets and formation of ice crystals.

**Table 9:** Freeze-thaw cycle.

Duration (Days) Nanoemulsions	1 (5°C)	2 (RT)	3 (5°C)	4 (RT)	5 (5°C)	6 (RT)
**Opt-VCO**	Stable	Stable	Stable	Stable	Stable	Stable
**VCOCP**	Stable	Stable	Stable	Stable	Stable	Stable

RT = Room Temperature.

The changes in particle size at temperature 25°C and 45°C for the VCO nanoemulsion containing copper peptide (VCOCP) were investigated over 90 days of storage time and the results are as depicted in Fig 6. Particle size of VCOCP remained almost constant at 25°C but showed slight changes at higher temperature (45°C) after 90 days storage time. Ribeiro *et al*. (2015) [38] observed significant changes in the particle size of cosmetic nanoemulsion at temperature 45°C. According to Ngan *et al*., (2014) [39], sample storage at high temperature (45°C) led to a higher kinetic energy in the Brownian motion of the oil droplets which could speed up their movement and collision. Despite the changes in particle size at temperature 45°C, VCOCP remained homogenous after 90 days storage period. Sample storage at elevated temperatures will increase the movement and collision between the oil droplets thus leading to droplets coalescence. The physical stability of Opt-VCO and VCOCP at storage temperatures of 25°C and 45°C for a period of 90 days is depicted in Table 10. All samples were able to maintain the homogeneity up to 90 days even at 45°C. The incorporation of xanthan gum enhances the viscosity of the bulk phase and reduces the probability of droplets collision, hence protecting the emulsion against coalescence [40].

**Fig 6:** Particle size changes (90 days) of VCOCP which was stable at 25°C and 45°C.

**Table 10:** Storage stability.

Day (s)	1		30		60		90	
Temperature (°C)	25	45	25	45	25	45	25	45
**Opt-VCO**	√	√	√	√	√	√	√	√
**VCOCP**	√	√	√	√	√	√	√	√

## 4. Conclusions

A three layers genetic algorithm neural network was applied for the modeling and processing of experimental data obtained from the preparation of VCO nanoemulsions for the prediction of particle size. The developed model was evaluated statistically and found out to have good prediction ability. The RMSE, R^2^ and ADD for the training and testing set were 5.7036, 0.9989, 2.6171 and 0.5902, 0.9973, 0.356 respectively. Xanthan gum content was the most dominant factor controlling the particle size followed by T80:PF68, VCO and water. The actual and predicted particle size values for the optimum formulations were 122.70 and 124.16 nm respectively. Most importantly, the particle size values of the optimum formulation showed no significant difference when compared to the particle size in the formulation containing the copper peptide. Zeta potential analysis and stability results indicated excellent physical stability of the final formulations and the products may find use in the cosmeceutical industry.
